# A Novel Algorithm for Breast Mass Classification in Digital Mammography Based on Feature Fusion

**DOI:** 10.1155/2020/8860011

**Published:** 2020-12-22

**Authors:** Qian Zhang, Yamei Li, Guohua Zhao, Panpan Man, Yusong Lin, Meiyun Wang

**Affiliations:** ^1^School of Computer Science, Zhongyuan University of Technology, Zhengzhou 450007, China; ^2^School of Information Engineering, Zhengzhou University, Zhengzhou 450001, China; ^3^Collaborative Innovation Center for Internet Healthcare, Zhengzhou University, Zhengzhou 450052, China; ^4^School of Software, Zhengzhou University, Zhengzhou 450002, China; ^5^Hanwei IoT Institute, Zhengzhou University, Zhengzhou 450002, China; ^6^Department of Radiology, People's Hospital of Zhengzhou University, Zhengzhou 450003, China

## Abstract

Prompt diagnosis of benign and malignant breast masses is essential for early breast cancer screening. Convolutional neural networks (CNNs) can be used to assist in the classification of benign and malignant breast masses. A persistent problem in current mammography mass classification via CNN is the lack of local-invariant features, which cannot effectively respond to geometric image transformations or changes caused by imaging angles. In this study, a novel model that trains both texton representation and deep CNN representation for mass classification tasks is proposed. Rotation-invariant features provided by the maximum response filter bank are incorporated with the CNN-based classification. The fusion after implementing the reduction approach is used to address the deficiencies of CNN in extracting mass features. This model is tested on public datasets, CBIS-DDSM, and a combined dataset, namely, mini-MIAS and INbreast. The fusion after implementing the reduction approach on the CBIS-DDSM dataset outperforms that of the other models in terms of area under the receiver operating curve (0.97), accuracy (94.30%), and specificity (97.19%). Therefore, our proposed method can be integrated with computer-aided diagnosis systems to achieve precise screening of breast masses.

## 1. Introduction

Breast cancer ranks first in morbidity and mortality amongst all diseases that affect females [1]. Recent research from the International Agency for Research on Cancer indicates that the incidence of breast cancer in China is gradually increasing, with more than 300,000 women diagnosed with breast cancer every year [2]. Mammography is widely used in the early screening of breast cancer because of its high diagnostic sensitivity for small lesions [3].

For radiologists, the detection or interpretation of breast masses via digital mammography is a time-consuming task [4]. Computer-aided diagnosis (CAD) systems are utilized in breast cancer diagnosis to reduce the burden of reading digital mammography images on radiologists and improve their diagnostic efficiency. Amongst various breast abnormalities (e.g., masses, microcalcifications, architectural distortions, and asymmetry), breast masses are difficult to distinguish from similar backgrounds because of their variable size and low contrast, both of which affect the diagnostic results.

Images obtained from X-rays display various body postures or different imaging angles, and effectively identifying the texture to be measured at different angles is important when performing texture analysis on the mass [5]. Convolutional neural networks (CNNs) can directly extract objective features from images without relying on feature extraction and manual selection [6]. A persistent problem in current mammography mass classification via CNN is the lack of local-invariant features, which cannot effectively respond to geometric image transformations or changes caused by imaging angles. This challenge can only be alleviated by manually manipulating the image rotation to augment the dataset, which is not effective for fine rotation.

Image texture is defined as a function of the spatial variation in pixel intensity (grey value) [7]. Texture analysis can systematically characterize complex visual patterns. The maximum response (MR) filter bank used in our study can deal with the rotation invariance of local images [8]. Moreover, the MR filter bank can effectively capture slight changes in the texture of images. Learned representations based on the MR filter bank can precisely model multiscale and multidirectional information that is important for breast mass diagnosis. However, a single texture feature cannot describe deep image features.

In summary, the feature representations of these two approaches are integrated into a single model. A novel method harnessing the complementary ability of fused rotation-invariant filters and deep learning for breast mass classification is proposed in this work. The MR filter bank is convolved with the images to generate textons, which are then fused with the feature representation extracted by ImageNet pre-trained CNN. The discriminative ability of the rotation-invariant filter banks and deep learning features in classifying benign and malignant masses is tested. Direct fusion and fusion after reduction approaches are implemented to compare and select the best classification model for breast mass diagnosis.

The proposed method has the following advantages:

1. Given that body postures or imaging angles vary in mammography mass images, a rotation-invariant filter set is used to analyze the texture of mass images
2. This study is the first to harness the complementary discriminative power of rotation-invariant and deep learning representations for breast mass classification
3. The fusion after implementing the reduction approach can harness better the complementarity between two groups of features and markedly improve the performance of breast mass classification

## 2. Related Work

Texture analysis can systematically characterize complex visual patterns. Via this approach, suspected regions can be examined by analyzing texture features. Haralick et al. [9] proposed the method of grey level co-occurrence matrices (GLCM), which is extensively used in image recognition and classification. Da Rocha et al. [10] combined diversity indices with GLCM as a way of describing the texture of breast tissues. Through this combination, they obtained an accuracy of 88.31%. Abdalla et al. [11] adopted the GLCM to extract the texture features of images from the Digital Database for Screening Mammography (DDSM) and achieved an accuracy of 91.67%. Co-occurrence matrices are also the main tools for texture analysis. By combining two-dimensional discrete wavelet transform with matrices to extract features from mammographic images, Beura et al. [12] achieved an accuracy of 97.4%. Texton is an effective tool for texture analysis. It is usually obtained through a filter set-based feature extraction approach that characterizes various pixel relationships in a specific area of an image [13–15]. Acharya et al. [16] applied the MR filter bank to convolve with images to generate textons. This approach attained 96% accuracy, demonstrating the effectiveness of the textons generated by the MR filter bank for classifying breast datasets. However, this approach does not consider deeper image features. A single texture feature cannot fully describe deep image features. Furthermore, the settings of the initial parameters of these traditional methods heavily rely on experience.

With the rapid development of deep learning, convolutional neural networks (CNNs) can directly extract objective features from images without relying on feature extraction and manual selection [17]. A single deep learning model is effective in fields involved in disease diagnosis, such as radiology and ophthalmology [18]. A previous study reported that deep learning outperforms physicians in classifying benign and malignant breast lesions [19]. Carneiro et al. [20] showed that pre-trained deep learning models can be applied to medical imaging. An area under the curve (AUC) of 0.90 was achieved in various mammogram datasets (e.g., INbreast and DDSM). Qiu et al. [21] recognized features from breast images through CNN and max pooling concepts. A prior study implemented a CNN along with intensity information and a decision mechanism to classify breast masses [22]. The increasing availability of large medical datasets facilitates the satisfactory performance of CNNs in assisting breast cancer diagnosis [23–25]. However, CNNs cannot explicitly realize rotation invariance of local images and thus cannot effectively respond to geometric image transformations or changes caused by imaging angles.

Some researchers sought to develop a methodology that combines texture analysis and deep learning for feature extraction. Wang et al. [26] explored a breast CAD method based on feature fusion with CNN deep features, texture features, and density features. He et al. [27] established a classification model on the basis of extracted textures and deep CNN features for evaluating diagnostic performance on differentiating malignant masses. They proved that the deep learning classification model for breast lesions, which was established according to image texture characteristics, can effectively differentiate malignant masses. These fusion methods are merely simple extensions at the feature level, and they do not consider the characteristics of mammography mass images.

## 3. Materials and Methods

The framework of the proposed method in this work is shown in Figure 1. The MR filter bank is convolved with the images to generate textons, which are then fused with the feature representation extracted by ImageNet pre-trained CNN. Direct fusion and fusion after reduction approaches are implemented to compare and select the best classification model for breast mass diagnosis.

### 3.1. Learning Representation from Texton

Texton can be generated using a filter set-based feature extraction approach that characterizes various pixel relationships in a specific area of an image. In past decades, many effective filter banks, such as Leung–Malik [28], Schmid [15], and MR filters [8], have been used to generate textons. The current study uses the MR filter bank containing isotropic and anisotropic filters to produce a satisfactory response to directional textures. Several studies have indicated that the MR filter bank can obtain textons with powerful discrimination [7, 29].

#### 3.1.1. MR Filter Bank

The MR filter bank consists of 38 filters. As shown in Figure 2, six orientations at three scales exist for two oriented filters in the first and second derivatives, thereby forming 36 anisotropic filters. The two isotropic filters are the Gaussian and Laplacian of Gaussian (LOG) filters.

If *G* is a Gaussian kernel function, then the first and second derivatives Gaussian filter can be defined as

(1) $$\begin{array}{c} G^{\prime }=G_{x}\cos\;\theta +G_{y}\sin\;\theta .\\ G^{\prime \prime }=G_{xx}\cos^{2}\;\theta +G_{yy}\sin^{2}\;\theta -2G_{xy}\cos\;\theta \;\sin\;\theta . \end{array}$$

LOG can be defined as

(2) $$\begin{array}{c} \text{LOG}=\nabla^{2}G=G_{xx}+G_{yy\;}. \end{array}$$

The MR8 filter bank is used to achieve rotational invariance. It yields eight responses: six responses from the three scales for two filters and two responses from the Gaussian and LOG filters. Using the MR8 filter bank to convolve with the images reduces the 38 filter responses to 8. This step not only reduces the dimensionality of the responses but also implies rotation invariance. Compared with the traditional rotation invariance filter, the MR8 filter bank can calculate the statistical information of high-order symbiosis in the relevant direction. Such information can help distinguish textures that are visually similar to the mass in its surrounding area.

#### 3.1.2. Local Binary Pattern Extraction

After the MR8 filter bank is used to generate textons, the local binary pattern (LBP) is then employed to extract features. LBP is a simple method that can effectively describe local image features by quantifying differences between the grey value of the neighborhood and the central pixel [30]. The texture descriptor is rotation-invariant and is not affected by brightness fluctuations during recognition, which can avoid the variation caused by different angles or imaging times of the mammography images. LBP can be defined as

(3) $$\begin{array}{c} {\text{LBP}}_{P,R}\left(x_{c,}y_{c}\right)=\left\{\begin{array}{cc} \sum_{n=0}^{P-1}s\left(g_{n}-g_{c}\right), & U\left({\text{LBP}}_{P,R}\right)\leq 2,\\ P+1, & \text{otherwise,} \end{array}\right. \end{array}$$

where

(4) $$\begin{array}{c} s\left(x\right)=\left\{\begin{array}{cc} 1, & x\geq 0,\\ 0, & x<0, \end{array}\right. \end{array}$$

*P* is the number of equally spaced points on the circumference with radius *R*, *g*_*c*_  is the pixel intensity at the centre point, and *U*(LBP_*P*,*R*_)  is a measure of uniformity applied to calculate the number of 0–1 transformations (i.e., from 0 to 1 or vice versa). The working principle of LBP is illustrated in Figure 3. The pixel values on the circumference are compared with the central pixel value to generate a binary value of “0” or “1” to extract the local contrast information.

The MR8 filter bank is used for the convolution with the images; each filter generates eight filter responses. The LBP algorithm is then applied to extract 36-dimensional feature vectors from each filter response to obtain a texton-based feature representation. A total of 288 (36 × 8) dimensional features are extracted from each image.

### 3.2. Learning Representation from Deep CNN

Given that large-scale training for medical tasks cannot be performed because of the lack of a medical dataset, a pre-trained network is introduced in this study. The InceptionV3 network is applied to the deep feature extraction. The computational cost and memory requirements of this network are lower than those of Residual Neural Network 50, Visual Geometry Group Network, and other networks. The main feature of the inception architecture is the calculation of nonlinear weighted sum modules (*σ*(*Wx*)) in each layer, which can be defined as

(5) $$\begin{array}{c} \sigma \left(\sum_{j=1}^{M}w_{j}x_{j}+b\right), \end{array}$$

where *M* is the number of neurons in this layer, *w*_*j*_ ∈ *W*, *W* is the weight matrix, *x* is the input vector, *b* is the deviation term, and *σ*(·) is the activation function. The module uses factorization to decompose 5 × 5 convolutions into two 1D (1 × 5 and 5 × 1) and compress the input or the dimension of the output of the previous layer, thereby effectively reducing the complexity and computational cost of the model. The experiment verifies that the effect of using random initialization to retrain the weights in the network is not as good as that using the ImageNet pre-trained network. Hence, the ImageNet pre-trained InceptionV3 model is used as the feature extractor. To use the pre-trained weights for fine-tuning, we repeat the grey value matrix of the image in three different channels of RGB to match the input of the retraining architecture. We utilize cross-entropy as the objective function and set the learning rate to be less than the initial learning rate pre-trained by the ImageNet. This step ensures that the network will not completely forget the features learned from the original dataset. The last softmax layer of the network is removed and the 1024-dimensional feature vector extracted from the layer with the largest receptive field (i.e., previous layer of the classification layer, that is, pool5) is selected as the final output features. This layer includes all different learning modes in the previous layer and can obtain the features with a strong discriminatory ability for classification [17].

### 3.3. Fusing Texton and Deep CNN Features

The idea of feature fusion comes from the early information fusion field, which is used for multisensor fusion in military applications [31]. Feature fusion methods are widely used in image recognition to achieve feature complementation and address the shortcomings of a single feature vector [32]. Two fusion strategies are designed to determine how the complementary information of the two features can be utilized.

#### 3.3.1. Direct Fusion

The most direct way to fuse two sets of feature vectors is to use cascade fusion [33], which can be defined as

(6) $$\begin{array}{c} X_{F}=\left[X_{\text{MR}},X_{\text{CNN}}\right], \end{array}$$

where *X*_MR_ and *X*_CNN_ are the texton- and deep CNN-based feature vectors, respectively; *X*_*F*_ is the fusion feature vector; and  dim(*X*_*F*_)=dim(*X*_MR_)+dim(*X*_CNN_). As described in Sections 3.1 and 3.2, dim(*X*_MR_)=288 and dim(*X*_CNN_)=1024. The dimension of the deep CNN features is more than three times the feature vectors obtained from MR8. The classification may focus on the deep CNN features and ignore the supplementary information in the textons. Therefore, we design a fusion strategy after feature reduction.

#### 3.3.2. Fusion after Reduction

In this strategy, feature selection is performed on two sets of feature vectors before cascade fusion is executed. Random forest is used for feature selection, which can analyze complex interactive features and is extremely robust to noisy and redundant data [34, 35]. On the basis of the feature importance measurement method, which uses the classification accuracy of Out-of-Bag (OOB) [36], feature subsets are selected according to the sequential forward selection (SFS) method.

The feature importance ranking method based on the classification accuracy of the OOB can be expressed as follows.

If the feature dimension is *N*, then bootstrap is adopted to extract *M* datasets. *M* OOB datasets are also generated accordingly.

**Step 1 .**

*m*=1 initialized and a decision tree *T*_*m* _ is created on the training set.

**Step 2 .**

The classification accuracy of the mth OOB dataset *A*_*m*_^oob^ is calculated.

**Step 3 .**

The feature *x*_*i*_(*i*=1,2, ⋯, *N*)) is disturbed in the OOB dataset, and the accuracy *A*_*m*,*i*_^oob^ is recalculated.

**Step 4 .**

Steps 2 and 3 are repeated for *m*=2,3, ⋯, *M*.

**Step 5 .**

The importance of *x*_*i*_ is calculated using

(7) $$\begin{array}{c} D_{i}=\frac{1}{M}\overset{M}{\underset{m=1}{\sum }}\left(A_{m}^{\text{oob}}-A_{m,i}^{\text{oob}}\right). \end{array}$$

**Step 6 .**

It is sorted in descending order. A high feature ranking indicates high importance.

Fivefold cross-validation is used to select more effective features. Subsequently, the OOB dataset is utilized to obtain the rank of importance and calculate accuracy. The sorted set of results with the most satisfactory classification effect is then selected, and the optimal feature subset is obtained using the SFS method. Finally, the cascade fusion of the two sets of features is executed.

### 3.4. Classification

The classifier is used to determine the relationship amongst the sets of attributes to predict the possible attribution results [37]. After the classifier is trained, the test data are fed into the network to predict the category and evaluate the performance of the algorithm. The following classifiers are used to classify benign and malignant masses.

For the direct fusion, the softmax in InceptionV3 is used as the classifier and the fused feature as its input. A dropout is added to the classification layer to enhance the robustness of the network. The stochastic gradient descent is used to minimize cross-entropy cost function.

For the fusion after reduction, a support vector machine (SVM) is utilized to distinguish benign and malignant masses on the basis of low-dimensional features. SVM is a supervised machine learning method widely used in statistical classification and regression analyses [38]. This technique can identify the best compromise between learning accuracy and learning ability of a specific training sample. In this study, the SVM based on radial basis function (RBF) kernel is used, and the features fused after reduction are used as inputs to obtain the probability of classifying the masses as benign or malignant.

Algorithm 1 shows the workflow of the method proposed here.

## 4. Results and Discussion

### 4.1. Image Databases and Preprocessing

In our study, we utilized three digital databases for screening mammography images, namely, Curated Breast Imaging Subset of DDSM (CBIS-DDSM) [39], INbreast [40], and Mammographic Image Analysis Society (mini-MIAS) [41] to evaluate performance of the proposed method.

#### 4.1.1. CBIS-DDSM

The CBIS-DDSM dataset is the curated breast imaging subset of DDSM. It consists of 861 mass cases and full mammography images, including mediolateral oblique and craniocaudal views of mammograms (i.e., 912 benign and 784 malignant masses).

#### 4.1.2. INbreast

The INbreast dataset was created by the Breast Research Group, INESCPorto, Portugal. It contains images of 115 patients for a total of 410 images, including images of masses, calcifications, and other abnormalities. It contains a total of 112 masses (i.e., 36 benign and 76 malignant masses).

#### 4.1.3. Mini-MIAS

The mini-MIAS, which is provided by the Mammographic Image Analysis Society, London, UK, dataset contains 322 mammogram images obtained from 161 women. It contains a total of 70 available mass images (i.e., 40 benign and 30 malignant masses).

Given that the sample sizes of INbreast and mini-MIAS datasets are too small, we merge them into one dataset. Therefore, these three databases are divided into two groups for evaluating the proposed method (Table 1). To render the dataset suitable for the pre-trained network and reduce the running cost, we extract 300 × 300 patches centered at masses in the three databases to build our dataset. Next, an adaptive histogram equalization [42] is applied to balance the contrast. For CBIS-DDSM, similar to other medical image classification experiments, the affine transformation is used to rotate the images by 0°, 90°, 180°, and 270° and reflect them along the horizontal axes to augment the dataset and avoid overfitting. For INbreast and mini-MIAS, each mass patch is augmented by the aforementioned affine transformation, and then these four images are flipped from left to right to generate eight images for each patch as the second dataset. Finally, each dataset is split into training (60%), validation (10%), and test (30%) sets.

### 4.2. Experiment Settings

The MR8 filter bank is operated in MATLAB and convolve with the mass images to generate textons. The InceptionV3 model based on Keras is used to transfer the pre-trained weights from ImageNet to the mass dataset. Given that mammography mass images are vastly different from ImageNet images, we propose to fine-tune our models to adjust the features of the last convolutional blocks and make them more data-specific. We utilize stochastic gradient descent to fine-tune the network and set the initial learning rate to 10^−5^. We divide the initial learning rate by 10 each time the validation error stops improving. Moreover, to improve the results and avoid overfitting, we perform L2 regularization and dropout. When training the SVM model, we employ the train and validation sets to fine-tune the C parameter for the SVM classifier. After tuning the models and choosing the best hyperparameters, we train each final model by using a stratified fivefold cross-validation with all the data and evaluate each model's performance.

### 4.3. Evaluation Metrics

In the diagnostic results of medical images, accuracy (Acc), sensitivity (Sens), and specificity (Spec) are the commonly used objective evaluation metrics. The area under the receiver operating characteristic curve (ROC) (i.e., AUC score) is another important metric used to evaluate the performance of diagnostic results. These evaluation metrics are calculated as follows:

(8) $$\begin{array}{c} \text{Acc}=\frac{N_{R}}{N},\\ \text{Sens}=\frac{\text{TP}}{\text{TP}+\text{FN}},\\ \text{Spec}=\frac{\text{TN}}{\text{FP}+\text{TN}}. \end{array}$$

In benign and malignant mass classification, if the malignant mass is classified as malignant, then the result will be true positive (TP). The result will become true negative (TN) if the benign mass is classified as benign. Similarly, if the benign mass is classified as malignant, then the result will be false positive (FP), which will become false negative (FN) if the malignant mass is classified as benign.

The k-fold cross-validation [43] method is adopted to evaluate the performance of the proposed method. The evaluation metrics in this study are derived from the fivefold cross-validation method.

### 4.4. Results and Analysis

#### 4.4.1. Direct Fusion

*(1) MR8 Features Only*. First, an MR8 filter bank is built, and the filter responses are collected by convolving them with the images. Second, the LBP algorithm is used to extract the 36-dimensional feature vectors from each filter response. Finally, the 288-dimensional feature vectors based on MR8 are obtained and used to train the softmax classifier. Fivefold cross-validation is applied to evaluate the average performance of this classifier in benign and malignant mass classification. As shown in Table 2, the AUC score and accuracy obtained by the MR8 features for classification are 0.79 and 70.21%, respectively.

*(2) Deep CNN Features Only*. The average accuracy obtained by the InceptionV3 model by using the initial weight is 72.21%. When the ImageNet pre-trained InceptionV3 is used to extract the 1024-dimensional feature vectors and train the softmax classifier described in Section 3.4, the classification results demonstrated improvements. The results are shown in the third row of Table 2, where the AUC score is 0.87 and the accuracy is 79.34%.

*(3) Direct Fusion*. The two features are directly fused using the cascade fusion method to train the softmax classifier. The classification results in the fourth row of Table 2 indicate that the AUC score is 0.92 and the accuracy is 80.02%.

Although the classification results after direct fusion are slightly better than those after using a single feature, the accuracy is almost the same as that when only deep CNN features are applied. This finding might be attributed to the excessively large feature dimension of the fusion, and the feature dimension of deep CNN being more than three times the feature obtained from MR8. Therefore, the classifier prefers the information contained in the deep CNN features during the classification, which is why the fusion method after feature reduction is developed.

#### 4.4.2. Fusion after Reduction

Random forest and SFS are used to select the feature subsets from the two groups of features. The OOB dataset and fivefold cross-validation are implemented to obtain the importance ranking and select the best set of features for the classification results, respectively. A total of 47 dimensional features are obtained, where 17 are obtained from the feature representation based on MR8 and 30 are obtained from the deep CNN features. The fused features are then fed into the SVM classifier. To obtain an effective comparison of the classification results of the fused features, we train the same SVM classifier by using the two feature subsets. A comparison of the classification results before and after fusion is shown in Table 3. The AUC score and accuracy of the MR8 feature subset only are 0.89 and 80.42%, respectively, in classifying CBIS-DDSM mass images. By comparison, the AUC score and accuracy of the deep CNN feature subset only are 0.92 and 88.67%, respectively. After implementing the reduction strategy, the fusion reaches an accuracy of 94.30% and an average AUC of 0.97, an increase of 0.05 and 14.28%, respectively, compared with those of the direct fusion strategy. This result suggests that training the classifier with the fusion features after reduction can better harness the complementarity of these two sets of features.

Figures 4(a) and 4(b) show the ROC curves of the direct fusion and the fusion after reduction, respectively. The three different color curves in each picture reveal that the area under the yellow ROC curve is the largest, which represents the classification result using the fusion features. The curves also confirm that fusion after reduction can effectively combine the advantages of the two features, and the feature representation based on MR8 can provide supplementary information to facilitate the CNN in classifying benign and malignant masses.

We also construct the fusion after reduction approach on INbreast and mini-MIAS. The classification results are summarized in Table 3. The AUC and accuracy of training the classifier by using the MR8 feature subset only are 0.88 and 88.47%, respectively, which are slightly higher than those of the classification performance by using CNN features. This result is obtained because these two databases are too small despite the fact that we have already augmented the data. CNNs cannot obtain additional effective features from a limited database. In spite of the limited number of datasets, training the classifier with fusion features still improves the performance of the classifier (AUC is 0.93 and accuracy is 93.59%). This result suggests that our method can achieve high performance even when sample sets are small and image bases are heterogeneous.

Three other machine learning classifiers are used to verify the classification performance of the fused features after reduction.  Figure 5 shows the classification results by using k-nearest neighbor classifier (kNN), SVM based on linear function kernel (SVM-linear), and extreme gradient boosting (XGBoost). Fusion features improve classification performance under all three classifiers (AUC scores are 0.89, 0.93, and 0.96, respectively). The three classifiers reflect the superiority of the fusion features after reduction. The confusion matrices using XGBoost as displayed in Figure 6 indicate that the number of misclassified benign and malignant masses after fusion is substantially reduced. Specifically, the number of malignant masses incorrectly classified as benign is reduced by nearly half.

#### 4.4.3. Comparative Analysis

To prove the complementary capabilities of MR8 features for CNNs, we adopt two popular deep learning models, namely, ResNet50 and Efficient-B7, to replace the InceptionV3 model in our method. The structure and depth of these models are suitable for medical image classification tasks with few training samples. MR8 + ResNet50 and MR8 + EfficientNet-B7 represent the use of fusion after reduction approach for fusing both MR8 and deep CNN features. As shown in Table 4, the fused features improve the performance of ResNet50 (ACC and AUC increased by 5% and 0.02, respectively) and Efficient-B7 (ACC and AUC increased by 8.55% and 0.05, respectively). Therefore, the features obtained from the MR8 filter can effectively compensate for the shortcomings of CNNs in feature extraction.

Various methods have been devised for classifying benign and malignant masses. The best case achieved by the method proposed herein is further compared with that of some recently developed classification methods (Table 4). The performance of our method is superior to that of traditional textural analyses and other machine learning methods [44, 45]. The performance of two deep learning methods [46, 47] is also compared with that of our method. As shown in Table 4, these two methods achieve high sensitivity (98.00% and 93.83%). However, their specificity is substantially lower than that of our method, suggesting that they may misclassify more negative masses compared with our method. Overall, the performance of our method is better than that of these two deep learning-based approaches. Moreover, the performance of methods described in [10, 11], which integrate multiple features to classify benign and malignant masses, is slightly lower than that of our method. The results establish the superiority and robustness of our proposed method.

## 5. Conclusions

Body postures or imaging angles vary in mammography masses. Malignant and benign masses may show similar features. Hence, they can be difficult to differentiate. In this study, a novel method based on texton fusion and CNNs for extracting mass features and classifying benign and malignant masses is proposed. Two fusion strategies, namely, direct fusion and fusion after reduction, are employed to fuse texton-based feature representations with deep CNN features. Moreover, these fusion strategies are adopted to explore how the complementary discrimination ability of two groups of features can be applied to mass classification tasks. These strategies are tested on the public databases CBIS-DDSM, INbreast, and mini-MIAS. Results show that the fused features can provide useful supplementary information for extracting mass features via CNN. By comparison, the fusion after reduction approach can harness better the complementarity of features extracted from the MR8 filter and deep CNN. Thus, this approach can achieve an accurate classification of benign and malignant masses. Experimental results demonstrate that our method outperforms other state-of-the-art methods without pixel-level annotation. Given that our method does not require any user interaction, it can be easily integrated into CAD systems for breast cancer.

However, mammography images have many pathological classifications, such as microcalcifications and structural distortions. At present, although this method has achieved good results in the classification of benign and malignant masses, it has not been tested in classifing and diagnosing other pathological classifications. With the expansion of our database, we will be able to optimize our method for other pathological classifications of breast images.

## Figures and Tables

**Figure 1:** Proposed method framework for mammogram mass classification.

**Figure 2:** MR filter bank.

**Figure 3:** LBP.

**Figure 4:** ROC curves of direct fusion and fusion after reduction. (a) The ROC curve of the average performance using direct fusion approach. (b) The ROC curve of the average performance using fusion after reduction approach.

**Figure 5:** Heat map of AUC score under kNN, SVM-linear, and XG boost using fusion after reduction with CBIS-DDSM.

**Figure 6:** Confusion matrix obtained by XGBoost using fusion after reduction approach with CBIS-DDSM. (a) Only MR8 features. (b) Only deep CNN features. (c) Fusing MR8 and CNN after feature reduction.

**Algorithm 1:** Mammography mass benign-malignant classification algorithm.

**Table 1:** Digital mammogram dataset.

	Database	Number of benign images	Number of malignant images	Total number of images
1	CBIS-DDSM	912	784	1696
2	INbreast	36	76	182
	Mini-MIAS	40	30	

**Table 2:** Comparison of MR8 features, deep CNN features, and direct fusion with CBIS-DDSM.

Methods	AUC	Acc
MR8 features only	0.7974	0.7021
Deep CNN features only	0.8711	0.7934
Direct fusion of MR8 and deep CNN features	0.9204	0.8002

**Table 3:** Comparison of MR8 features, deep CNN features, and fusion after reduction.

Dataset	Methods	AUC	Acc
CBIS–DDSM	MR8 features only	0.8964	0.8042
	Deep CNN features only	0.9262	0.8867
	Fusing MR8 and deep CNN features	**0.9795**	**0.9430**

INbreast + mini–MIAS	MR8 features only	0.8812	0.8847
	Deep CNN features only	0.8553	0.8728
	Fusing MR8 and deep CNN features	0.9383	0.9359

**Table 4:** Comparison of proposed method with other mass classification methods.

Dataset	Methods	Sens	Spec	Acc	AUC
CBIS-DDSM	ResNet50	77.31%	82.07%	79.50%	0.86
	MR8 + ResNet50	83.17%	85.94%	84.50%	0.88
	EfficientNet-B7	80.47%	81.05%	80.75%	0.80
	MR8 + EfficientNet-+B7	89.88%	88.02%	89.30%	0.85
DDSM	M. Hussain et al. [44]	–	–	85.53%	0.87
BCDR	L. Fangyi et al. [45]	88.93%	93.41%	91.65%	0.96
INbreast	N. Dhungel [46]	**98.00%**	70.00%	90.00%	–
CBIS-DDSM	C. Yuanqin [47]	93.83%	92.17%	93.15%	0.95
DDSM	S. V. da rochaa [10]	85.00%	91.89%	88.31%	0.88
DDSM	Q. Abbas [11]	92.00%	84.20%	91.00%	0.91
CBIS-DDSM	Proposed method	89.97%	**97.91%**	**94.30%**	**0.97**

## Data Availability

The data used to support the findings of this study are available from the corresponding author upon request.
